This article has been retracted.

# On the Intelligent Computing Model of Diagnosis Teaching in Preschool Education in Colleges and Universities under the Background of Big Data

**DOI:** 10.1155/2022/7183032

**Published:** 2022-09-30

**Authors:** Xiaoqiong Ding

**Affiliations:** Yunnan College of Business Management, Kunming City, Yunnan Province 650032, China

## Abstract

In order to infer the cognitive state of students and provide teachers with the potential learning state of students, a diagnostic teaching model for preschool education in colleges and universities under the background of big data is proposed. By increasing students' programming ability and modeling students' theoretical and practical abilities at the same time, the cognitive diagnosis is introduced into the field of computer teaching, so as to make it applicable to computer classrooms and provide students' cognitive information needed for teaching. The experimental results show that the advantages of the CDF-CSE approach gradually emerge as the training data become sparse (the proportion of training data decreases from 80% to 20%). In the combined questions of the three datasets, when the training set is 20% and MAE is used as the criterion, the CDF-CSE model improves by 47.8%, 65.8%, and 49.8%, respectively, compared with the other methods that perform best on the training set. When the number of questions is small, the CDF-CSE model improves by 37.8%, 42.5%, and 27.7% on RMSE on three datasets, respectively, compared with the best-performing other methods. When there are more questions, it has 32.3%, 36.5%, and 45.6% improvement, respectively. It is concluded that this model can accurately predict students' performance in computer courses and provide detailed and rich cognitive reports.

## 1. Introduction

With the comprehensive popularization of Internet technology, the 21st century has entered an era of information explosion. Information technology has fully entered human social life, and informatization has become the general trend of the development of the current era [1, 2]. In this context, all walks of life have accumulated a large amount of available data, and it has become an inevitable trend to improve and upgrade related industries through the mining and application of these data. With the gradual advancement of informatization in the field of education, various intelligent teaching assistance platforms have emerged one after another. Due to their massive resources and learning characteristics independent of time and space, these teaching assistance platforms have developed rapidly and attracted a large number of users. At present, the intelligent teaching assistance system is gradually becoming a mainstream education method in the knowledge era, which has gradually become an ideal learning environment for learners to carry out collaborative learning, knowledge construction, and wisdom development. As a new type of modern education platform, the intelligent teaching assistance system has completed the transformation from “teacher-centered” to “student-centered.” On the one hand, the intelligent teaching assistance system is free from the constraints of time and space and has the advantages of autonomy and openness. On the other hand, the current teaching assistance system is still based on the knowledge-infusion teaching method, similar to traditional education, which is composed of learning materials.

At present, the research on educational assistive technology for educational examination data has attracted the gradual attention of researchers in the fields of education and data mining, but the current educational assistive technology still faces great challenges [3]. On the one hand, effective educational assistance is based on adequate and accurate understanding of students, that is, a comprehensive analysis of students' learning ability and cognitive level is required. Therefore, student modeling has become an important direction and research basis of educational auxiliary algorithms. On the other hand, on the basis of student modeling, intelligent auxiliary technologies for the educational process should also be studied and improved, such as the automatic construction of collaborative learning groups and the prediction of students' performance trends, as shown in Figure 1.

## 2. Literature Review

Miulescu et al. developed a cognitive diagnosis model of disciplinary knowledge ability based on the Bayesian model test method. The purpose of using the cognitive diagnosis model was to achieve different results according to the DINA model data for different structures. Differentiation between items could also be analyzed using this method. A likelihood function was established between item level and correlation [4]. Qin et al. pointed out that a diagnostic assessment of a person's cognitive processes, processing skills, and knowledge structure was often referred to as cognitive diagnosis or cognitive diagnostic assessment. Cognitive diagnostic assessments were used to measure individual-specific knowledge structures (knowledge structures) and processing skills (processing skills) [5]. Qiu et al. believed that cognitive diagnostic tests should test at least three users' cognitive characteristics [6]. The first was that the user had significant knowledge and skills in a specific cognitive domain. However, this knowledge and capabilities could be achieved at a higher level. And the second was the basic structure of knowledge, which could indicate that the user could use some skills to carry out the knowledge construction. The third was the cognitive process of users. In summary, the cognitive diagnosis was based on traditional measurement theory, but it emphasized that test measurement must thoroughly examine the subject's internal mental processes [7]. Xu et al. believed that the cognitive diagnosis model could be simply divided into two parts, namely, generalized cognitive diagnosis and narrow cognitive diagnosis [8]. The generalized diagnosis mainly indicated the observation of user scores and the internal characteristics of users, which could not only be used to construct psychological theories but also be used in education and teaching. Cognitive diagnosis in a narrow sense refers to classifying subjects according to whether they have mastered the skills or characteristics tested in the fields of education and teaching, mainly to achieve better communication between teachers and students. Daghestani et al. used a visual method to display the results of cognitive diagnosis to more intuitively display the student's diagnosis report [9]. Prada et al. used a cognitive diagnostic model to evaluate students' ability to master knowledge points and make personalized test item recommendations [10]. Bhat et al. found that there was a large amount of data on MOOCs related to knowledge points. Therefore, they tried to extract features from various types of materials such as texts and teaching videos on MOOCs and proposed a method based on representation learning for the first time (representation learning-based method) to automatically infer the learning order between knowledge points in MOOCs [11]. In addition to machine learning methods, Chang et al. turned their attention to information theory to formulate an information-theoretic view of knowledge point prerequisite relationships and automatically construct relationships between concepts from text corpora, so as to generate reading lists for studentsto help them learn the relevant material in the best way [12].

In the research study, the students' programming abilities were modeled based on a probabilistic graphical model, and cognitive diagnosis was introduced into the field of programming education. At the same time, the students' theoretical level and practical ability were modeled. By using the same knowledge points that appear in theoretical questions and experiments, the two capabilities were linked for a more comprehensive diagnostic report.

## 3. Research Methods

### 3.1. Problem Definition

Now, defining our problem, we assumed that there are a total of *M* students, *K* knowledge points, *N*_*i*_ questions, and *N*_*e*_ experiments. *R* is a score matrixof *M* rows and *N*_*i*_ columns. And *R*_*ji*_ represents the *j*student's scores on the *ith* question, where *j* ∈ {1,…, *M*}, *i* ∈ {1,…, *N*_*i*_}, *R*_*ji*_ ∈ [0,1]. For programming experiments in the course, *R*_*je*_′ indicates the *j* student's scores on the experiment *e*, where *e* ∈ {1,…, *N*_*e*_}, *R*_*je*_′ ∈ [0,1]. The matrix *Q* indicates the knowledge points contained in each topic, with a total of *N*_*i*_ rows and *K* columns. *q*_*ik*_indicates whether the topic contains *k* knowledge points, where *k* ∈ {1,…, *K*}. The matrix indicating the knowledge points contained in each experiment is denoted as *Q*′, with a total of *N*_*e*_ rows and *K* columns. *q*_*ek*_ indicates whether the experiment *e* contains *k* knowledge points. Under normal circumstances, *q*_*ik*_=1 means that the topic *i* requires *k* knowledge points, and zero is the opposite. The meaning of *q*_*ik*_ is similar. In the model, the matrix *Q* is normalized, such that ∑_*k*=1_^*K*^*q*_*ie*_=1, ∑_*k*=1_^*K*^*q*_*ke*_′=1.

*R*, *R*′, *Q*, *Q*′ are known. Our goal is to give students' cognitive assessment in computer teaching, which is divided into the following three aspects [13].

1. Diagnose *j* student's programming ability *c*_*j*_
2. Give *j* student the theoretical mastery *α*_*jk*_ of *k* knowledge point and the corresponding practical application ability *β*_*jk*_
3. Predict the *j* student's answers *η*_*ji*_ to new theoretical question *i* and the practical status *η*_*je*_′ of experiment *e*, where *α*_*jk*_, *β*_*jk*_ ∈ (0,1), 0 means no mastery and 1 means complete mastery

The specific application process of cognitive diagnosis in computer course teaching: First, students pass exams or homework, answer theoretical questions, or write codes. Teachers or teaching assistants give a specific score according to the students' answers. The cognitive diagnostic model uses these scores, along with other teaching information, to make inferences about students' abilities and generate cognitive reports that are returned to students. Students can carry out the targeted training based on cognitive reports to check and fill gaps [14].

### 3.2. Cognitive Diagnosis Model

#### 3.2.1. Cognitive Diagnosis Model

*(1) Code Capability*. To assess students' coding ability, we refer to the research findings in educational psychology. Everyone has a high-order latent characteristic that indicates a general ability to learn a subject. In the model, in order to represent the practice level of students, the high-level latent feature is visualized as a parameter that each student *i* has to represent the student's programming learning ability *c*_*j*_. This parameter is not for a certain knowledge point, but for the embodiment of his own programming ability [15]. In Layman's terms, each student *j* has an independent parameter *c*_*j*_ that represents the student's ability to write programs. The programming ability *c*_*j*_ and the student's theoretical knowledge level together determine the corresponding level of the code written by the student.

*(2) The Mastery and Application of Knowledge Points*. *α*_*jk*_ is recorded as the *j* student's ability to use knowledge point *k* to solve theoretical problems, and at the same time, *β*_*jk*_ is recorded as the ability of *j* student to use knowledge point *k* to write code. In the model, it is reasonably assumed that there is no direct correlation between the various abilities, that is, the abilities of a student in different skills do not affect each other, and the abilities of different students are independent of each other. According to the experience gained in the past teaching process, the two abilities of the same skill are related. Students can apply it only after they have mastered the skill theoretically. Therefore, a hypothesis is proposed.

The *j* student's ability to program using knowledge point *k* is proportional to the student's theoretical mastery of the knowledge point and basic coding ability, i.e., *β*_*jk*_=*c*_*j*_*α*_*jk*_.

That is to say, it is believed that a person's ability to use knowledge point *k* to program depends on his theoretical level of the corresponding knowledge points, which is limited by his basic programming ability.

*(3) The Degree of Mastery of the Topic*. *η*_*ji*_ is used to indicate the student's mastery of a theoretical question, and *η*_*je*_′ is used to indicate the student's mastery of an experiment. The traditional cognitive diagnosis model considers that a student's mastery of a topic is related to the knowledge points that the student has learned and the knowledge points needed to answer the question. In practice, each topic contains one or more knowledge points [16]. If the student answers the question completely or gives a partial answer, it means that the student has used the specific knowledge points required by the question, and it is recognized that the student has mastered or partially mastered the corresponding knowledge points. Based on the above analysis, we define students' mastery of the problem as the following assumptions.

The degree of master of a student *j* on topic *i* is related to the level of the student's mastery of the knowledge points examined by the topic, that is, the degree of master of the student on the topic *η*_*ji*_=∑_*k*=1_^*K*^*α*_*jk*_*q*_*ki*_ and the degree of mastery of the student in the *e* experiment *η*_*je*_′=∑_*k*=1_^*K*^*β*_*jk*_*q*_*ke*_′.

In short, a student's score on a certain question is proportional to the student's mastery of the knowledge point examined in the question. The more proficient the student at playing the knowledge point, the better his performance in the question that includes the knowledge point.

*(4) Actual Score*. In actual situations, due to mistakes or guesswork, students may give some correct answers without mastering the knowledge points or write wrong answers due to subjective factors such as being careless for a while, resulting in a slight deviation between the actual score and the actual mastery degree [17]. So, it is necessary to take into account the impact of these factors on students' final scores in the model. Therefore, refer to the method of probability matrix decomposition in the recommendation system, that is, there is a certain gap between the score predicted by the model and the user's actual score on the item, and this gap conforms to the Gaussian distribution. Therefore, the actual score is simulated according to the students' mastery of the problem as given in the following formulae:

(1) $$\begin{array}{c} R_{ji}∼N\left(\eta_{ji},\sigma_{R}^{-1}I\right)\text{,} \end{array}$$

(2) $$\begin{array}{c} R_{je}^{\prime }∼N\left(\eta_{je}^{\prime },\sigma_{R^{\prime }}^{-1}I\right)\text{.} \end{array}$$

*σ*_*R*_ and *σ*_*R*′_ are the hyperparameters and **I** is the identity matrix. In our model, the actual score follows a Gaussian distribution with the mean value of the mastery level, that is, the actual score should be related to the students' mastery of the problem. However, some external factors will lead to the probability of deviation.

*(5) Summary*. In order to understand the abovementioned methods better, the proposed model is summarized as the probability graph, in which the gray circles are the observed values and the white circles are the unknown quantities. It can be seen from the figure that the observable value is the *M*students' performance *R* on the *N*_*i*_ questions and *R*′on the*N*_*e*_ experiments, as well as the matrix *Q* and *Q*' of the corresponding relationship between each question and *K* knowledge points. The mastery of degree {*α*_*jk*_}_*k*=1_^*K*^ of each student *j* in each knowledge point *k* corresponds to a programming level {*β*_*jk*_}_*k*=1_^*K*^. *α*_*jk*_, and *c*_*j*_ determine *β*_*jk*_. The student's *j* master degree *η*_*ji*_ on question *i* is determined by the student's master's degree{*α*_*jk*_}_*k*=1_^*K*^ and the knowledge point {*q*_*ki*_}_*k*=1_^*K*^ investigated by the topic, and student's *j* code master's degree *η*_*je*_′ on experiment *e* is determined by the knowledge point coding ability {*β*_*jk*_}_*k*=1_^*K*^ and the knowledge point {*q*_*ke*_′}_*k*=1_^*K*^ investigated by the experiment question. Finally, the actual scores of student *j* on question *i* and experiment *e*, *R*_*ji*_ and *R*_*je*_′, are affected by the degree of master's {*α*_*jk*_}_*k*=1_^*K*^ and {*β*_*jk*_}_*k*=1_^*K*^, respectively [18]. Following the setting of the HO-DINA model, our parameters obey the prior distribution of the following formulae:

(3) $$\begin{array}{c} c_{j}∼N\left(\mu_{c},\sigma_{c}^{-1}I\right)\text{,} \end{array}$$

(4) $$\begin{array}{c} \alpha_{jk}∼N\left(\mu_{\alpha },\sigma_{\alpha }^{-1}I\right)\text{.} \end{array}$$

In formulae (3) and (4), *σ*_*c*_ and *σ*_*α*_ are the hyperparameters.

#### 3.2.2. Parameter Optimization

According to the above probability graph and the assumed prior of parameters, we can obtain the posterior distribution of *c* and *α*, as shown in the following formulae.

(5) $$\begin{array}{c} p\left(c,\alpha \;|\;R,R^{\prime }\right)\propto p\left(R\;|\;\alpha \right)p\left(R^{\prime }\;|\;c,\alpha \right)p\left(c\right)p\left(\alpha \right)\text{.} \end{array}$$

In formula (5),

(6) $$\begin{array}{c} p\left(R_{ji}\;|\;\alpha_{j}\right)=N\left(\overset{K}{\underset{k=1}{\sum }}\;\alpha_{jk}q_{ki},\sigma_{R}^{-1}I\right)\text{,} \end{array}$$

(7) $$\begin{array}{c} p\left(R_{je}^{\prime }\;|\;c_{j},\alpha_{j}\right)=N\left(\overset{K}{\underset{k=1}{\sum }}\;c_{j}\alpha_{jk}q_{ke}^{\prime },\sigma_{R^{\prime }}^{-1}I\right)\text{,} \end{array}$$

(8) $$\begin{array}{c} p\left(c_{j}\right)=N\left(\mu_{c},\sigma_{c}^{-1}I\right)\text{,} \end{array}$$

(9) $$\begin{array}{c} p\left(\alpha_{jk}\right)=N\left(\mu_{\alpha },\sigma_{\alpha }^{-1}I\right)\text{.} \end{array}$$

Taking the negative logarithm of the posterior distribution, the following formula can be obtained.

(10) $$\begin{array}{c} F\left(c,\alpha \right)=\frac{\sigma_{R}}{2}\overset{N}{\underset{j=1}{\sum }}\;\overset{N_{i}}{\underset{i=1}{\sum }}\;{\left(R_{ji}-\eta_{ji}\right)}^{2}+\frac{\sigma_{R^{\prime }}}{2}\overset{M}{\underset{j=1}{\sum }}\;\overset{N_{e}}{\underset{e=1}{\sum }}\;{\left(R_{je}^{\prime }-\eta_{je}^{\prime }\right)}^{2}+\\ \frac{\sigma_{\alpha }}{2}\overset{M}{\underset{j=1}{\sum }}\;\overset{K}{\underset{k=1}{\sum }}\;{\left(\alpha_{jk}-\mu_{\alpha }\right)}^{2}+\frac{\sigma_{c}}{2}\overset{M}{\underset{j=1}{\sum }}\;{\left(c_{j}-\mu_{c}\right)}^{2}+C\text{.} \end{array}$$

In formula (10), *C* is a constant, *f* is our loss function, and our goal is to minimize the error function *F*(*c*, *a*).

Next, the way to optimize our parameters is introduced. The optimization process is mainly divided into two steps, and the detailed process is as follows:

*(1) Step 1 Optimize*. *α*. It is fixed and each student's ability to answer each question is independent of each other, that is, *α*_*jk*_ are independent of each other, which means that the whole parameter optimization can be decomposed into multiple independent parts, and optimize each part of *α*_*jk*_ in parallel to improve the efficiency of the algorithm [19]. In the research, the gradient descent method was used to optimize a single part, and the following formula is obtained:

(11) $$\begin{array}{c} \alpha^{new}=\alpha^{ol\;d}-r_{1}\frac{\partial }{\partial \alpha }F\left(c,\alpha \right)\text{.} \end{array}$$

In formula (11), *α*^*ol* *d*^ is the parameter before the update, *α*^*new*^ is the parameter after the update, *r*_1_ is the learning rate, and *∂*/*∂αF*(*c*, *α*) is the partial derivative of the function *F*(*c*, *α*) on *α*.

(12) $$\begin{array}{c} \frac{\partial }{\partial \alpha }F\left(c,\alpha \right)=-\sigma_{R}\overset{N_{i}}{\underset{i=1}{\sum }}\;q_{ki}\left(R_{ji}-\eta_{ji}\right)-\sigma_{R^{\prime }}\overset{N_{e}}{\underset{e=1}{\sum }}\;c_{j}q_{ke}^{\prime }\left(R_{je}^{\prime }-\eta_{je}^{\prime }\right)+\sigma_{\alpha }\left(\alpha_{jk}-\mu_{\alpha }\right)\text{.} \end{array}$$

*(2) Step 2 Optimize*. *c*. Similarly, *α* is fixed and each student *j*'s parameters *c*_*j*_ are independent of each other, so the gradient descent method is used to optimize each *c*_*j*_ simultaneously, as shown in the following formula.

(13) $$\begin{array}{c} c^{new}=c^{ol\;d}-r_{2}\frac{\partial }{\partial c}F\left(c,\alpha \right)\text{.} \end{array}$$

In formula (13), *c*^*ol* *d*^ is the parameter before the update, *c*^*new*^ is the parameter after the update, *r*_2_ is the learning rate, and *∂*/*∂cF*(*c*, *α*) is the partial derivative of the function *F*(*c*, *α*) on *c*.

(14) $$\begin{array}{c} \frac{\partial }{\partial c}F\left(c,\alpha \right)=-\sigma_{R^{\prime }}\overset{N_{e}}{\underset{e=1}{\sum }}\;\left(R_{je}^{\prime }-\eta_{je}^{\prime }\right)\left(\overset{K}{\underset{k=1}{\sum }}\;\alpha_{jk}q_{ke}^{\prime }\right)+\sigma_{c}\left(c_{j}-\mu_{c}\right)\text{.} \end{array}$$

According to formulae (11) and (13), the value of the sum is iteratively updated, and the abovementioned process is only stopped when the model converges or the number of iterations reaches a certain number of times [20]. Finally, the algorithm outputs the students' cognitive parameters and the students' basic coding ability, and we can make predictions about the students' grades based on these two parameters.

### 3.3. Experiment

#### 3.3.1. Experimental Data

To validate the proposed model, the preschool data of students in a computer course at a university were collected to validate our model. The collected real-world datasets were organized, cleaned, and formatted, excluding some special data, such as the data of students who barely handed in homework. Our experiments were conducted on two real datasets (data from the computer courses “Data Structure” and “Network Security”) and a simulated dataset, all three datasets containing students' theoretical *R* and experimental grades *R*′, as well as questions and the knowledge examined in the experiment *Q* an d *Q*′. In the real dataset, the students' grades and the knowledge points required by the topic were provided by teachers or teaching assistants [21]. The basic situation of the dataset is given in Table 1.

*(1) Course “Data Structures” Dataset*. The first dataset is the student practice data collected in the course “Data Structure,” containing 96 students, 58 theoretical questions, and 10 experimental questions, a total of 6528 pieces of data. The course contains a total of 19 knowledge points, including common concepts of data structures such as “find,” “graph,” and “binary tree.” Theoretical questions are mainly theoretical investigations of this knowledge. While, experiments include classical implementations of various algorithms as well as simulated real-world scenarios, such as “bank queues” and “flight reservations” [22].

*(2) Course “Network Security” Dataset*. The second real dataset is a dataset collected from the course “Network Security,” which contains 10 theoretical questions answered by 194 students and 8 experimental answers, a total of 3492 pieces of data. The course contains a total of 7 knowledge points, involving “encryption/decryption,” “buffering,” and so on. The content of the experiment includes “shell-code” and “vulnerability” and other related content.

*(3) Simulation Dataset*. Finally, a simulated dataset is constructed. In the simulated dataset, we set up 1000 students, 200 theoretical questions, 50 experiments, and a total of 250,000 pieces of data. The dataset contains a total of 20 knowledge points.

First, the theoretical questions are taken as an example to introduce how to simulate students' answering situations [23]. In order to simulate the different skill levels of different students, each student is assigned a personalized personal model. Assuming that the students' mastery of knowledge points obeys the Gaussian distribution, the students' ability determines the mean and variance of the personal model. For students with a higher degree of mastery of knowledge points, the mean of the personal model is higher; while for students with a low degree of mastery of knowledge points, the mean of the personal model is correspondingly lower. At the same time, the variance of the model corresponding to the careful student is smaller, that is, the student's score can better reflect his true level. Relatively, the variance of the personal model corresponding to the careless student is larger because his answering situation may not be stable. In addition, matrix *Q* is generated to link questions and knowledge points together. The students' answers to each question are generated based on the student' personal model and the knowledge points contained in the questions indicated by the matrix *Q*. To reflect the instability of the students' on-the-spot performance, a random error in the range [−0.1, 0.1] is added to the simulated scores. If the error value is negative, it means that the student does not play at their true level; if it is positive, it means that the student has played well or guessed part of the answer. Finally, our simulated scores range between [0, 1], and even after adding the error value, it will not exceed this range.

A similar method is used to simulate the experimental performance of students. A student's practical ability on a certain knowledge point is related to the student's theoretical mastery. Therefore, to simulate the students' practical ability, a random number in the range [0, 0.1] is subtracted from the students' theoretical ability. This ensures that the students' practical ability is linked to their theoretical ability. But in order to conform to the actual situation, the students' practical ability will not exceed their theoretical mastery of knowledge points. Finally, students' scores on experimental questions are simulated by using the method described above.

#### 3.3.2. Experimental Settings

Compared with the four methods, the validity of the proposed cognitive diagnosis model is proved.

*Item Response Theory (IRT).* IRT is a classical cognitive diagnostic method, which models students' potential abilities and characteristics of questions.

*Probability Matrix Factorization (PMF).* PMF is a latent factor model that projects students and questions into a low-dimensional space.

*FuzzyCDF.* This method introduces the concept of fuzzy sets, regards the student's performance as a continuous value, and combines a variety of classical cognitive diagnosis methods to improve itself.

*NeuralCD.* This approach combines deep learning and remains interpretable.

Mean absolute error (MAE) and root mean square error (RMSE) are used to evaluate the performance of each model. During the training of CDF-CSE, when the parameters do not change (the difference between the results of two consecutive iterations is less than 10^−10^), the training is stopped and the results are obtained. For each experiment, it runs 100 times, and the results are averaged. It is worth mentioning that the IRT model and FuzzyCDF are implemented using the MCMC method. In the experiments of these two algorithms, the number of iterations is set as 10000, and sample parameters are obtained based on the results of the last 2500 iterations. To make a fair comparison, the parameters are adjusted to record the best performance of each algorithm. Finally, all algorithms are implemented in Python and run on Windows 10 machines with 8 GB of memory and an i5 3.2 GHz CPU.

## 4. Result Analysis

### 4.1. Score Prediction

First, the accuracy of each model in predicting students' scores is compared to judge whether the cognitive results given by the model are reliable. Parameters *α* and *β* are the theoretical and practical abilities of students given by the model. These two parameters are used to predict students' scores, and the cognitive results obtained by each method are tested by the error between predicted scores and real scores. In the experiment, different implementations of matrix decomposition methods, namely, PMF-5D, PMF-10D, and PMD-KD were used as PMFS with 5, 10, and *K* (knowledge point number) potential factors, respectively.

First, the fixed training set accounted for 80%, and the test set accounted for 20%. In the dataset containing both theoretical and experimental data, the performance of each model is compared.  Table 2 shows the experimental results for predicting student performance. Overall, CDF-CSE performance is the best among the three datasets because it can establish a correlation between theory and practice [24]. It is worth mentioning that NeuralCD uses a deep learning method, which requires a large number of instances for training, so it performs poorly on the two smaller datasets and performs well on the larger simulated datasets, but it is still not as good as CDF-CSE.

In order to observe the performance of different datasets in different levels of sparse levels, a training set of different sizes is constructed, with 10%–80% of each candidate's scoring data, and the rest are for the tests. Since the NeuralCD is poor in small datasets, it is not compared in this experiment. In addition to the model of the NeuralCD, the models will be compared to the dataset that contains the theoretical problem, the dataset that contains only the experimental problem, and the performance of the dataset that contains two types of data. From the different angles mentioned above, the overall comparison is different. Figures 2(a)–2(f), 3(a)–3(f), and 4(a)–4(f) show the results of the CDF-CSE and other methods in three different datasets. In the results of the empirical research, it is observed that the CDF-CSE performs best in all datasets.

Specifically, it outperforms PMF in terms of combining teaching assumptions, outperforms IRT in terms of quantitatively analyzing students, and outperforms all other methods in terms of combining theory and experimentation. In addition, the parameters obtained by CDF-CSE can directly represent the cognitive state of students inferred by the model, which is interpretable. However, the parameters obtained by IRT and PMF cannot give students' abilities in various knowledge points. Such a model, even if it can accurately predict students' scores, has little effect in diagnosing students' cognitive status. More importantly, as the training data become sparser (the proportion of training data drops from 80% to 20%), the advantages of the CDF-CSE method gradually emerge. For example, in the comprehensive question of three datasets, when the training set is 20% and MAE is used as the judging criterion, CDF-CSE is improved by 47.8%, 65.8%, and 49.8% compared with other methods that perform best on the training set.

Obviously, CDF-CSE is more accurate than other methods because the CDF-CSE method can be trained on datasets with two different problems, theoretical and experimental. That is, compared with other models that only consider one kind of problem, CDF-CSE can obtain more information during the training process. For the dataset containing two types of problems, the model will provide different probability assumptions for the two kinds of problems. This matches the actual situation. Even in the special case where the probability distribution of students' scores on both questions is the same, CDF-CSE can be trained normally. However, other models can only consider one probability distribution, which inevitably produces errors. In other words, on different types of questions that examine the same knowledge points, students' performance should be the same, and CDF-CSE makes full use of this feature. When the model observes that students have a good grasp of a knowledge point in theory, the model reasonably predicts that the students can use the knowledge point well in practice. At the same time, we can also infer the theoretical level of students according to the situation of students in the experiment. This approach is in line with the actual teaching experience, and the experimental results also prove the feasibility of the method. In contrast, other models do not do this, so they occasionally perform poorly on some datasets. And compared with other models, the assumptions of CDF-CSE are also more applicable to subjective questions and computer teaching, which also leads us to achieve good performance on all three datasets.

To sum up, CDF-CSE can capture the characteristics of students more accurately, and it is also more suitable for practical teaching scenarios with sparse data.

### 4.2. Course Process Follow-Up

Furthermore, we hope that cognitive diagnostic models can not only evaluate students after the course is completed but also provide feedback to students as the course progresses. In this way, the cognitive diagnosis model can help students understand their own cognitive structure in the learning process and timely check and fill in gaps to improve learning efficiency. Therefore, the process of taking a class is simulated, and experiments are carried out in the process. In the experiment, a dataset containing two kinds of questions is used, and the data volume of the training set is fixed at 80%, and the rest is used as the test set. At the same time, according to the chronological order, only a small number of questions are used for training at the beginning, and the number of questions is gradually increased after getting the results.

CDF-CSE still performs the best on all datasets. It performs well in the early stages (when there are few knowledge concepts and questions). Its advantages gradually become apparent as the amount of data increases. For example, when the number of items is small, the CDF-CSE model achieves 37.8%, 42.5%, and 27.7% improvement in the RMSE metric on the three datasets, respectively, compared with the other best-performing methods. Improvement. It has 32.3%, 36.5%, and 45.6% improvement when the number of questions is large.

The result proves that the method of combining theoretical and experimental performance to analyze the cognitive state of students is still feasible in the case of little data. Even in the early stages of teaching, CDF-CSE can use more information than other models to better analyze the characteristics of students. As the course develops, the analysis results are gradually more accurate. To sum up, the proposed CDF-CSE can well follow up the whole process of computer course teaching.

## 5. Conclusions

According to the experimental results, the CDF-CSE method is superior to other methods in predicting student performance. This is because CDF-CSE can extract common features from two types of questions and at the same time can distinguish the differences between them, so as to diagnose students' theoretical cognition and practical ability. Compared with other models, CDF-CSE is more suitable for teaching computer courses, and the results given are more abundant and accurate. The experimental results also confirm that our model can be applied to different situations. Therefore, more comprehensive cognitive information can be analyzed using different data from students. From the experimental results, it is concluded that CDF-CSE can solve the problem of inaccurate feedback of traditional cognitive diagnostic models in computer course teaching and provide more detailed and interpretable cognitive analysis results. In computer science teaching courses, such results help teachers understand the teaching situation and can also help students learn in a targeted manner.

## Figures and Tables

**Figure 1:** Auxiliary education model.

**Figure 2:** The performance of each model on the “data structure” course datasets. (a) Data structure-theoretical-MAE. (b) Data structure-theoretical-RMSE. (c) Network security-experimental-MAE. (d) Network security-experimental-RMSE. (e) Data structure-mix-MAE. (f) Data structure-mix-RMSE.

**Figure 3:** Performance of each model on the “network security” course datasets. (a) Network security-theoretical-MAE. (b) Network security-theoretical-RMSE. (c) Network security-experimental-MAE. (d) Network security-experimental-RMSE. (e) Network security-mix-MAE. (f) Network security-mix-RMSE.

**Figure 4:** Performance of individual models on simulation datasets. (a) Synthetic-theoretical-MAE. (b) Synthetic-theoretical-RMSE. (c) Synthetic-experimental-MAE. (d) Synthetic-experimental-RMSE. (e) Synthetic-mix-MAE. (f) Synthetic-mix-RMSE.

**Table 1:** Dataset overview.

Dataset	Number of students	Knowledge points	Number of theoretical questions	Number of programming questions	Data volume
“Data structure”	96	19	58	10	6528
“Network security”	194	7	10	8	3492
“Simulation dataset”	1000	20	200	50	250000

**Table 2:** Experimental results for predicting student performance.

Model	“Data structure”		“Network security”		“Simulation dataset”	
	MAE	RMSE	MAE	RMSE	MAE	RMSE
IRT	0.358 ± 0.02	0.415 ± 0.02	0.203 ± 0.02	0.247 ± 0.02	0.227 ± 0.02	0.327 ± 0.02
PMF-5D	0.316 ± 0.02	0.380 ± 0.02	0.195 ± 0.02	0.246 ± 0.02	0.212 ± 0.02	0.265 ± 0.02
PMF-10D	0.319 ± 0.02	0.383 ± 0.02	0.196 ± 0.02	0.248 ± 0.02	0.219 ± 0.02	0.265 ± 0.02
PMF-KD	0.319 ± 0.02	0.383 ± 0.02	0.196 ± 0.02	0.248 ± 0.02	0.213 ± 0.02	0.265 ± 0.02
FuzzyCDF	0_283 ± 0.01	0.376 ± 0.02	0_210 ± 0.01	0.230 ± 0.02	0.220 ± 0.01	0.314 ± 0.02
NeuralCD	0.464 ± 0.03	0.481 ± 0.02	0.429 ± 0.02	0.498 ± 0.02	0.120 ± 0.02	0.235 ± 0.02
CDF-CSE	0.147 ± 0.01	0.231 ± 0.01	0.066 ± 0.01	0.146 ± 0.01	0.106 ± 0.01	0.132 ± 0.01

## Data Availability

The labeled datasets used to support the findings of this study are available from the corresponding author upon request.
